The article "Correlation of Carotid Artery Intima-Media Thickness with Calcium and Phosphorus Metabolism, Parathyroid Hormone, Microinflammatory State, and Cardiovascular Disease" was retracted in 2024. Reasons: signs of a paper mill; suspected computer-generated content; unreliable results or conclusions; concerns about the data.

# Correlation of Carotid Artery Intima-Media Thickness with Calcium and Phosphorus Metabolism, Parathyroid Hormone, Microinflammatory State, and Cardiovascular Disease

**DOI:** 10.1155/2022/2786147

**Published:** 2022-03-12

**Authors:** Peng Huang, Junhua Tan, Xianjun Gu, Meiying Huang, Feifan Huang, Ruiying Ma, Jie Wang

**Affiliations:** Department of Nephrology, The Affiliated Hospital of Youjiang Medical University for Nationalities, Baise, 533000 Guangxi, Guangxi Zhuang Autonomous Region, China

## Abstract

The internal thickness of the carotid artery is the vertical distance between the intima of the carotid artery and the middle mold. Its normal thickness is less than 1 mm. It can be used to judge the degree of arteriosclerosis. Under normal circumstances, the change of the internal thickness of the carotid artery is caused by cardiovascular disease. The purpose of this article is to study the relationship between the thickness of the carotid artery and the metabolism of calcium and phosphorus, parathyroid hormone, microinflammatory state, and cardiovascular disease. This article uses ultrasound measurement to measure the IMT of ESRD patients and carotid arteries with normal renal function. The analysis includes blood pressure, blood phosphorus, blood calcium, blood creatinine, blood urea nitrogen, blood sugar, glycosylated hemoglobin, blood lipids, parathyroid hormone, and C reaction. The correlation between clinical indicators includes protein and carotid IMT in ESRD patients which can be used in designing a diagnostic plan for patients through correlation research. The results showed that the carotid artery IMT of ESRD nondialysis patients was 13% thicker than that of those with normal renal function, and it was significantly positively correlated with age, blood pressure, blood phosphorus, glycosylated hemoglobin, and C-reactive protein. The correlation ratio with calcium and phosphorus was about 0.1.

## 1. Introduction

Insufficient carotid artery thickness can easily lead to disorders of calcium and phosphorus metabolism, abnormal secretion of bone metabolism indicators such as window hormones, leading to fibroosteitis, bone dysplasia, osteomalacia, and other bone diseases with poor prognosis. Abnormal bone metabolism refers to a series of diseases such as osteoporosis and osteomalacia that are caused by a series of pathological factors that lead to problems in bone metabolism. Changes in CIMT are often considered to be associated with cardiovascular disease risk, but very few studies have reported this correlation. The aim of this paper is to investigate the correlation of carotid intima-media thickness with calcium and phosphorus metabolism, parathyroid hormone, microinflammatory status, and cardiovascular disease in patients. The KDIGO guidelines define CKD-MBD caused bone disease induced by disorder of mineral metabolism [1]. Due to renal failure, patients with Maintenance Hemodialysis(MHD) have higher iPTH (Immunoreactive parathyroid hormone), resulting in less bone formation than bone resorption, increased bone loss of cortical bone and carcinogenic bone, and a significant increase in the risk of vertebral body and local fractures [2]. Since iPTH has a good histological connection with ROD, it has been widely used in the diagnosis of bone and kidney diseases in the past [3]. However, for patients with low vitamin D3 levels (and other patients with low iPTH levels), the result of the iPTH test is the sum of 1-84PTH and 7-84PTH. The latter causes a decrease in blood calcium and competes with 1-84PTH. Comparing the biological activity of PTH1-84 and iPTH can better clarify bone transport in MHD patients [4]. Therefore, if the indicators with strong specificity and high sensitivity to CKD-MBD can be found from the detection indicators, the combination of iPTH is of great significance for the timely prevention and diagnosis of CKD-MBD [5].

The carotid intima-media thickness (CIMT) is a reliable marker of subclinical atherosclerosis and cardiovascular events [6]. Until today, no studies have investigated whether epicardial adipose tissue (EAT) is more important for CIMT and atherosclerotic plaques, and epicardial adipose tissue is a substitute for lipid accumulation or circulating lipids in special visceral tissues [7]. The Kocaman SA study used a cross-sectional and prospective observational design and included 252 hospitalized patients, Figure 1 shows the variation of CIMT mean value with EAT [8]. EAT is determined as an anechoic space under the pericardium on two-dimensional echocardiography and is measured perpendicular to the front of the free wall of the right ventricle at the end of systole [9, 10]. EAT is significantly correlated with CIMT. With the increase of EAT thickness, CIMT increases significantly (for patients with EAT is less than 5 mm) [11]. Multiple linear regression analysis showed that age (Beta: 0.406), male (Beta: 0.244), and EAT (Beta: 0.450) were independent related factors of CIMT [12]. However, such experiments are not stable, and the result data obtained will not be very accurate [13, 14].

The occurrence of cardiovascular disease is related to the consumption of vegetables. Epidemiological studies have shown that the risk of eating vegetables is inversely proportional to the risk of cardiovascular disease [15]. Guo-Yi et al. have studied the ingredients of vegetables. Vegetables have great potential for preventing and treating cardiovascular diseases [16]; vitamins, essential ingredients, dietary fiber, plant protein, and phytochemicals are biologically active ingredients. The cardioprotective effects of vegetables may involve antioxidant effects [17]. Anti-inflammatory, antiplatelet properties regulate blood pressure, blood sugar, and blood lipid levels; reduces myocardial damage; and regulates related enzyme activities, gene expression, and signal transduction pathways, and other biomarkers related to cardiovascular disease [18, 19]. In addition, several vegetables and their biologically active ingredients have been proven to prevent cardiovascular disease in clinical trials [20]. However, the composition of vegetables is variable, which reduces the accuracy of the results [21].

The innovation of this article lies in the domestic and foreign research on the correlation between CIMT and acyclic plaque formation and coronary heart disease [22], comparing the correlation and difference between bilateral CIMT and coronary artery disease [23]. CIMT can not only reflect the occurrence and severity of coronary artery disease but also reflect the number of blood vessels in coronary artery disease, and it can also reflect the degree of vascular stenosis. The degree of effect of the intervention on CIMT progression predicts the degree of CVD risk reduction. These data support the use of descending CIMT progression as a surrogate marker of CVD risk. CIMT has specific reference value for the diagnosis of coronary heart disease [24]. Combining the patient's baseline condition and carotid artery, Doppler ultrasound can improve the diagnostic accuracy of coronary heart disease, but due to the limitations of Doppler ultrasound itself, it is necessary to find a more objective and accurate diagnosis method; the degree of sensitivity, specificity, and accuracy of Doppler ultrasound in the diagnosis of occupying thyroid lesions is significantly higher than that produced by conventional, but in the clinic, ultrasound elastography discrimination is experienced and technology needs to be improved to further improve the accuracy [25].

## 2. Materials and Methods

### 2.1. Experimental Materials

83 cases of ESRD nondialysis patients were selected for long-term treatment in the Department of Neurology of our hospital, 45 males and 38 females, including 52 cases of chronic seminogenic nephritis, 18 cases of diabetic renal failure, 8 cases of ischemic renal failure, Langchuang 3 cases of nephritis, 2 cases of polycystic kidney disease.

Inclusion criteria are as follows: 18 years of age or older, diagnosed with chronic renal failure (uremia); without renal replacement therapy, no infection, surgery, blood transfusion, and heart failure. Within a short period of time, there was no pregnancy, breastfeeding, severe malnutrition or other serious diseases. All selected patients have been informed of their consent and voluntarily participate in this study.

Exclusion criteria are as follows: age less than or equal to 18 years old, primary hyperthyroidism, acute renal failure, window edema, poisoning, combined malignant tumors, active immune tissue diseases, liver failure such as hepatitis and cirrhosis, blood system diseases, congenital heart disease, and abnormal blood coagulation mechanism.

At the same time, 50 patients with normal renal function treated in our hospital from December 2016 to April 2020 were randomly selected, including 24 males and 26 females, including 31 cases of renal syndrome, 9 cases of chronic spirochetal nephritis, and IgA with renal function. There were 5 cases of failure, 3 cases of diabetic renal failure, and 2 cases of purple kidney.

### 2.2. Data Collection Method

To further investigate the factors influencing carotid intima-media thickness, the carotid IMT measurement is as follows: The patient is placed in a supine position with the neck completely exposed. Siemens S3000 ultrasonic diagnostic instrument was used, the probe frequency is 4-8 MHz, starting from the proximal end of the bilateral joint carotid artery, measuring the vertical distance between the hospitals without obvious points, the internal connection of the block, the average value and the risk interface, and the average value after three measurements. The average bilateral IMT thickness is the IMT value of the patient's carotid artery. The blood count was collected the next morning the patient was admitted to the hospital. Blood calcium (Ca), blood phosphorus (P), blood creatinine (Cr), fasting venous blood, blood urea nitrogen, blood glucose (GLU), glycosylated hemoglobin (HbA1c), protein C (CRP), total cholesterol (TCH), and high-density lipoprotein (HDL) levels are detected by an automatic biochemical analyzer. Electrochemical photometric determination of serum parathyroid hormone (PTH) level. After a 15-minute break in the morning, all patients used a standard mercury pulse monitor to measure blood pressure in their right arm.

### 2.3. Ultrasound Inspection Methods

To find out the carotid intima-media thickness of patients, use cervical ultrasound to evaluate carotid artery calcification. All the patients were checked by a permanent ultrasound recorder in our hospital, but he did not know the patient's condition. The subject was asked to place his position and detector on the outside of the trachea in front of the neck. Measure the thickness of the center of the carotid artery 1 cm below the artery and vagina, and observe the longitude and lateral two-dimensional images in real time.

ITM refers to the subsonic gray area not shown on the arterial column, the vertical distance from the middle of the material yard to the interface between the middle and the outer mold. The average value of the bilateral ITM is used as the patient's ITM value. The judging criteria are as follows: the common carotid artery IMT is greater than or equal to 1.0 mm, that is, the carotid artery calcification plate is formed. Thickening of the median carotid artery, or the absence of carotid plate and carotid plate. This is the so-called carotid artery calcification process. If the artery wall extends into the official cavity, the longitudinal and lateral images and thickness of the same part become thicker than others. Half of the neighboring area is called atheroma.

### 2.4. Carotid Artery Intima-Media Thickness Measurement Experiment

The CIMT measurement site is the left and right common carotid arteries, 10 mm from the carotid sinus, left and right common carotid arteries. During the measurement, the subject was asked to turn the head of the No. 45 ship to the other side and place it underwater. Each subject underwent the same experienced ultrasound examination and repeated the measurement three times. The instrument used is the same ultrasound system, which is equipped with an L9-3mhz ultrasonic sensor and standard image settings. In epidemiology and clinical practice, the measurement of CIMT should take into account the gender, age, and ethnic differences of subjects. Due to the lack of uniform diagnostic criteria for carotid dysplasia worldwide, China defines the common carotid artery as greater than or equal to 1.0 mm or carotid sinus greater than or equal to 1.2 mm, and the coefficient of variance is less than 2.9%.

### 2.5. Statistical Methods

All statistical data should use the Chinese version of the SPSS 19.0 software. The measurement data is represented by the average value and standard deviation, and the measurement data is represented by the composition ratio. The analysis of variance was used to compare the average values between multiple measurement groups, and the LSD method was used to compare the differences between the groups. The X2 test is used to compare the differences between the measured data sets. Classification and inspection shall be adopted for the grade data. Correlation analysis adopts Pearson's correlation analysis. *P* < 0.05 indicates that the difference is statistically significant.

## 3. Results

### 3.1. Correlation Analysis of Carotid Artery Intima-Media Thickness and Calcium and Phosphorus Metabolism

In general, among the 7000 health checkups, there are 4000 males and 3000 females; age 23-86 years old, with an average age of 50 years. There are 1 400 patients with phosphate and potassium metabolism disorder, including 1 200 males and 200 females. The prevalence of phosphate and potassium metabolism disorder in the study population is 20.7%; the prevalence of phosphate and potassium metabolism disorder in men (30%) is significantly higher than the prevalence of female phosphorus and potassium metabolism disorder (7%). Calcium and phosphorus metabolism refers to the entire process of calcium and phosphorus being taken up by the body in food, then synthesized and broken down in the body, and finally excreted. Calcium in the body comes mainly from food and is mostly absorbed in the upper part of the small intestine. The effect of carotid artery IMT was analyzed by covariance. The carotid IMT of the phosphate and potassium metabolism disorder group before correction was significantly higher than that of the nonphosphate and potassium metabolism disorder group; Carotid IMT was higher in the corrected phosphorus and potassium metabolism disorder group than in the precorrected phosphorus and potassium metabolism disorder group. After adjusting for factors such as gender and age, the phosphorus and potassium metabolism, the carotid IMT of the disordered group was still higher than the IMT of the nonphosphate and potassium metabolism disordered group. The comparison of carotid artery IMT values before and after correction is shown in Figure 2:

Phosphorus and potassium metabolism disorder is a situation where the metabolic risk factors of a variety of cardiovascular diseases are concentrated in one person. The factors of phosphorus and potassium metabolism disorders are more complex, not only related to the environment, but also to genetics. The factors of phosphorus and potassium metabolism disorders may be due to poor nutrition and electrolyte disorders in the body caused by irregular life and diet all the time. Need to pay more attention to the diet, it is usually best to exercise properly ,have a regular diet, and promote blood flow. The barriers to phosphorus and potassium metabolism are caused by complex genetic and environmental factors. Therefore, the main problem is insulin resistance and high insulin. Both can cause and accelerate atherosclerosis by causing hypertension and disorders of glucose and lipid metabolism.

### 3.2. Correlation Analysis between Carotid Artery Intima-Media Thickness and Parathyroid Hormone

Parathyroid hormone (PTH) is a basic single-chain polypeptide hormone secreted by the main cells of the parathyroid glands. Its main function is to regulate the metabolism of calcium and phosphorus in vertebrates, resulting in an increase in blood calcium levels and a decrease in blood phosphorus levels. The serum OC, iPTH, and blood phosphorus concentrations of the parathyroid group were higher than those of the control group, and there were statistical differences (*P* < 0.05). The blood calcium concentration was lower than that of the control group, and the parathyroid group was higher than the control group. As shown in Table 1:

In the parathyroid hormone group, OC and iPTH were significantly positively correlated. The specific data are shown in Figure 3:

Through analysis, it can be observed that the serum OC and iPTH levels of the parathyroid hormone group were significantly higher than those of the non-MHD group, the blood phosphorus concentration was significantly higher than that of the non-MHD group, and the Ca concentration was lower than the control group, but the difference was statistically significant. The renal function of patients with uremia was severely damaged, the filtration rate of the pellet was lower than 16 ml/min, and the serum OC level was higher than that of the control group. According to research, changes in serum osteocalcin usually occur when GFR is less than 20 ml/min, and osteocalcin is mainly excreted from the kidneys. After renal dysfunction in MHD patients, the level of iPTH increases, renal clearance decreases, and iPTH deposition in the kidney decreases. The half-life is prolonged. There are high levels of iPTH in the body.

### 3.3. Correlation Analysis of Carotid Artery Intima-Media Thickness and Microinflammatory State

Intravascular inflammation due to the involvement of inflammatory substances is called microinflammatory state. Dialysis patients do not have systemic or local overt clinical signs of infection, but there is a low-level, persistent inflammatory state, manifested by elevated inflammatory factors. It is generally accepted that the microinflammatory response is the result of sustained activation of the monocyte/macrophage system, and that hemodialysis patients can suffer from monocyte activation due to contact between peripheral blood monocytes and contaminated endotoxin in the dialysis membrane or dialysis fluid, which can exponentially exacerbate the development of the inflammatory response. According to the CCA-IMT value measured by B-ultrasound, the study subjects were divided into 5 groups, namely, 0.60 mm group, 0.80 mm group, 0.90 group, 1.20 group, and larger than 1.20 mm group. There was no statistical difference in age, gender, height, body weight, body mass index, systolic blood pressure, diastolic blood pressure, fasting blood glucose, hemoglobin, smoking history, and drinking history among individuals in each group.  Figure 4 shows the comparison of serum hsCRP, ferritin, ALB, pre-ALB, and TF between groups. It can be seen from the figure that the contents of clear hsCRP and ferritin increased with the increase of CCA.IMT value, showing a positive correlation (*r* is 0.84 and, respectively, 0.89); ALB, pre.ALB, and TF content decreased with the increase of CCA.IMT value, showing a negative correlation (*r* is -0.62, -0.78, and -0.65, respectively).

Atherosclerosis is a chronic vascular proliferative inflammation, and inflammation plays an important role in its occurrence. Serum inflammation index occurs at different stages of atherosclerosis. C-reactive proteins are mainly acidic phase proteins produced in the liver. Usually trace amounts can be seen in normal human serum. C-reactive protein plays a regulatory role by activating complement and enhancing phagocytosis to remove invading pathogenic microorganisms and damaged, necrotic, and apoptotic tissue cells in the plasma when the body is infected or damaged by tissue (acute protein).

Specific and nonspecific inflammatory stimuli can be significantly increased. It is not only an index of clinical inflammation serum but also has the effect of inflammatory factors, directly participating in the main stages of atherosclerosis and promoting the development of atherosclerosis. On the one hand, the formation of atherosclerosis is accompanied by an increase in plasma protein C reaction; on the other hand, C-reactive protein may promote the occurrence of atherosclerosis. Inflammatory factors enter the vascular endothelium from macrophages to regulate the expression of adhesion factors and regulate the arterial wall. In cells and circulation, the role of single-cell proinflammatory factors is ancient, further promoting the formation of atherosclerosis. Therefore, C-reactive protein is actually a preinflammatory factor related to the occurrence and development of atherosclerosis.

### 3.4. Correlation Analysis of Carotid Artery Intima-Media Thickness and Cardiovascular Disease

Cardiovascular disease is a collective term for cardiovascular and cerebrovascular diseases and refers to ischemic or hemorrhagic diseases of the heart, brain, and systemic tissues caused by hyperlipidemia, blood viscosity, atherosclerosis, and hypertension. Comparison of CIMT and clinical indicators in CVD cardiovascular patients are as follows: the age, LDL, CRP, and CIMT of CVD cardiovascular patients are significantly higher than those of patients without CVD, while the Alb and Mg of patients are significantly lower than those of HD patients without CVD, as shown in Figure 5:

According to the accounting analysis of 90 HD patients regression, the HD-related risk factor combined with cardiovascular disease is CIMT. CIMT is a powerful predictor of cardiovascular disease. CIMT and CRP are related, and both are related to cardiovascular events. The risk factor CIMT is closely related to stroke and myocardial infarction. Hypomagnesemia is a risk factor for patients with carotid atherosclerosis. Mg is closely related to vascular calcification and atrom arteriosclerosis and has an obvious negative relationship with CIMT. Hypomagnesemia can worsen the patient's arteriosclerosis. Together, they increase the incidence of cardiovascular disease. Therefore, the LDL, CRP, and CIMT of HD patients with cardiovascular disease increased significantly, and the blood concentration of Alb and Mg decreased significantly. Risk factors for cardiovascular disease are related to CIMT and hypomagnesemia. Correcting hypomagnesemia in HD patients and improving carotid arteriosclerosis are important means to prevent cardiovascular disease in HD patients.

According to the characteristics of physical ultrasound, the distance between the two parallel rays between the inner ridge and the middle of the carotid artery is called the thickness of the middle heart artery. Fatigue is the initial stage of the carotid artery which is a sign of atherosclerosis. As a manifestation of systemic atherosclerosis, carotid atherosclerosis has a pathological basis similar to coronary arteries and cerebral arteries. Therefore, the increase in the thickness of endothelial arteries is closely related to the occurrence of cardiovascular and cerebrovascular diseases.

### 3.5. Analysis of Influencing Factors of Carotid Artery Intima-Media Thickness

#### 3.5.1. Association Analysis of Serum igG and CIMT

According to the analysis results, the serum IgG level is generally negatively correlated with the prevalence of CIMT thickening. With the increase of IgG concentration, the prevalence of CIMT thickening showed a downward trend, and there was no significant difference between men and women. As an immune disease, whether it is fungal immunity or cellular immunity, it is achieved by affecting deposition, the absorption, and peroxidation of oxidized low-density lipoprotein in the formation of atherosclerosis. Unsaturated fatty acids are fatty acids that constitute body fat and are indispensable to the human body. Insufficient unsaturated fatty acids in the diet can easily produce the following diseases: an increase in LDL and LDL cholesterol in the blood, producing atherosclerosis, and inducing cardiovascular and cerebrovascular diseases. There is evidence that the increase in serum IgG is related to the formation of lesions and the decrease in serum cholesterol levels. Low-density lipoprotein contains a large amount of multipotential unsaturated fatty acids. These fatty acids undergo peroxidation under the action of excessive free radicals and reagents and finally produce low-density lipoprotein modified by malonylurea. Studies have shown that the degree of AS is positively correlated with MDA-LDL. MDA-LDL is a clinical risk factor for AS, that is, T cells can secrete a large amount of AS and a large number of IgG anti-MDA-LDL antibodies, thereby delaying the development of AS.

#### 3.5.2. Association Analysis of Parathyroid Glands and CIMT

The incidence of secondary hyperthyroidism in dialysis patients is higher. High levels of window-specific hormones affect the deposition of calcium and phosphorus, leading to vascular calcification, a mineral and bone disease associated with CKD. Analysis shows that high window hormones can promote the level of inflammatory factors and the proliferation of smooth muscle vascular cells. Parathyroid hormone can also directly increase the composition of FGF23 by activating the PTH-R1 receptor and indirectly stimulate the composition of potassium triol. The renal tubule 1a is hydroxylated, and the above mechanisms are involved in and accelerate the occurrence of vascular calcification. In addition, the relationship between parathyroid hormone and vascular calcification was studied using endothelial cells and detected by Western blot and ELISA methods. Western blot is a current method for semiquantification of proteins in combination with internal reference, which can reflect the information of molecular weight, and ELISA can quantify certain proteins and hormones. It was found that BMP-2 labeled osteoblasts were exposed to 10^10 mmol/l PTH. The differentiation effect is the greatest. The expressions of osteogenic proteins BMP 2 and BMP 4 increase. Parathyroid hormone is believed to promote the differentiation of endothelial cell osteoblasts, mainly through protein-labeled extracellular 1/2 kinase pathway and nuclear factor kB pathway, but at present, the effects of PTH on the differentiation of endothelial cells and bone fibers and its mechanism have not been fully elucidated, and further research is needed.

#### 3.5.3. Association Analysis between Inflammation and CIMB

Through analysis, it can be known that the main reason for the microinflammation of dialysis patients is the low immune function of dialysis patients, which may be accompanied by anemia, release of uremic toxin, and other reasons to promote the development of inflammation. These inflammatory factors mainly include C-reactive protein, tumor necrosis factor, interleukin-1, interleukin-6, and insulin growth factor. They activate the bone formation process in different ways and promote vascular calcification. Recently, in order to confirm the role of inflammation in vascular calcification, experimental rats were divided into rats with kidney damage and rats with inflammation with kidney damage. Rats were injected with adenine into the stomach and measured the level FGF23 mRNA, which confirmed that inflammation not only directly stimulates vascular calcification but also indirectly promotes the occurrence of vascular calcification in dialysis patients by increasing the level of FGF23. In addition, the exposure of macrophages to calcium phosphate mediators was also studied, and it was found that macrophages can promote inflammation-promoting release factors through protein kinase pathway C and RANKL, which may also promote macrophages to release inflammatory factors and promote vascular calcification. These confirmed related inflammation and vascular calcification.

## 4. Discussion

The CIMT value studied in this paper reflects not only the number of coronary artery disease but also the severity of coronary artery disease and the degree of vascular stenosis. CIMT has certain reference value for the diagnosis of coronary heart disease. Combining the basic condition of the patient's carotid artery and Doppler ultrasound can improve the accuracy of the diagnosis of coronary heart disease, but due to the limitations of Doppler ultrasound itself, it is necessary to find a more objective and accurate diagnosis method.

This article analyzes that the disease is a known risk factor for atherosclerosis and vascular disease and is associated with increased mortality. Inflammatory mediators activate blood calcification pathways, leading to upregulation of bone transformation-related factors. TNF-*α*, IL-6, and IL-1b can cause phenotypic changes of vascular smooth muscle cells. In CKD patients, the increase of inflammatory mediators is related to arterial calcification. In animal studies, inflammation promotes blood calcification and bone loss in mice and acts through the factor kB (NF-*κ*B) pathway. In in vitro experiments, long noncoding RNA-ANCR reduced the expression of Runx2 and BMP-2 in vascular smooth muscle cells by inhibiting the activation of NP-KB.

This article analyzes the sporadic increase in calcium and calcium load caused by the use of active vitamin D in the urea population, active vitamin D receptor antagonists, and calcium-phosphorus binders. The abnormal ossification of vascular smooth muscle cells on high calcium medium may be due to the secondary increase of phosphate transferred to the cells. L-type calcium channels are also involved in the process of vascular calcification. In vitro inhibition of verapamil type I calcium channels can reduce the occurrence of vascular calcification. In addition, Norin can also reduce calcification in VSMC medium. High levels of extracellular calcium are related to the release of stratigraphic cysts and may promote cell death and release, both related to the progression of calcification.

## Figures and Tables

**Figure 1:** Variation of CIMT mean value with EAT.

**Figure 2:** Comparison of carotid IMT values before and after correction.

**Figure 3:** Scatter plot of OC and iPTH.

**Figure 4:** Comparison of serum between groups.

**Figure 5:** Comparison of CIMT between two groups of cardiovascular patients.

**Table 1:** Comparison of the parathyroid hormone group and normal control group.

Group	OC (pg/ml)	iPTH (pg/ml)	Ca (mmol/L)	P (*μ*mol/L)
Parathyroid hormone group	103.3	331	2.16	1.67
Normal control group	6.3	48.06	2.24	1.05
t	-7.8	-7.6	-2.4	-7.3
P	0	0	0.1	0

## Data Availability

The data used to support the findings of this study are included within the article.
